RETRACTED

# The Effect of Social Cognitive Interaction Training on Schizophrenia: A Systematic Review and Meta-Analysis of Comparison with Conventional Treatment

**DOI:** 10.1155/2022/3394978

**Published:** 2022-08-16

**Authors:** Yan Tang, Linhua Yu, Dongyang Zhang, Fang Fang, Zhaoxia Yuan

**Affiliations:** ^1^Department of Psychiatry, Affiliated Mental Health Center & Hangzhou Seventh People's Hospital, Zhejiang University School of Medicine, Hangzhou, Zhejiang 310013, China; ^2^Department of Emergency, Affiliated Mental Health Center & Hangzhou Seventh People's Hospital, Zhejiang University School of Medicine, Hangzhou, Zhejiang 310013, China

## Abstract

**Background:**

Existing antipsychotic medications may alleviate the majority of patients' symptoms, but they have no discernible impact on improving social function and quality of life. Psychotherapy is required for the treatment of schizophrenia. However, contemporary psychotherapy technology intervention techniques are limited to a single intervention, and there is a lack of holistic and complete intervention approaches. Social cognition and interaction training is a comprehensive therapy strategy that has been employed in clinical practice; however, the therapeutic efficacy has been inconsistently reported. As a result, we included controlled clinical trials for meta-analysis in order to carefully assess the efficacy of this therapy.

**Methods:**

This meta-analysis searched all RCT literatures related to social cognitive interaction training (SCIT) published before April 2022 and assessed the effect of this method in the treatment of schizophrenia. The data in the literatures were combined, and the standardized mean difference (SMD) and mean difference (MD) with 95% confidence interval (95% CI) were calculated to predict the negative symptom score, positive symptom score, PANSS score, and social function score of the patients after treatment.

**Results:**

14 RCT studies including 1167 inpatients with schizophrenia were included in this study using a retrospective observational study method, including 590 patients treated with SCIT and 577 patients treated with treatment as usual (TAU). The pooled analysis showed that patients after SCIT had lower negative symptom scores (SMD = −1.66, 95% CI (-2.32, -1.00), *P* < 0.0001), lower positive symptom scores (MD = −4.03, 95% CI (-7.69, -0.36), *P* = 0.03), lower PANSS total scores (MD = −6.33, 95% CI (-12.43, -0.23), *P* = 0.02), and higher social functioning scores (SMD = 0.77, 95% CI (0.34, 1.20), *P* < 0.001) than those after TAU.

**Conclusion:**

Our findings support that SCIT is helpful to improve the relief of symptoms and the improvement of social function in patients with schizophrenia, providing a basis for the application of SCIT in hospitalized patients and community patients, and can guide the treatment and intervention of patients with schizophrenia.

RETRACTED

## 1. Introduction

Schizophrenia is a common chronic persistent disease in psychiatry, which is characterized by high disability rate and high recurrence rate [1]. The condition is characterized by severe cognitive impairment, which may affect patients' social functions such as self-care, daily living, communication, and family life and significantly diminish their quality of life [2]. Existing antipsychotic drugs can relieve most of the symptoms of patients but have no significant effect on the improvement of social function and quality of life of patients, and the side effects of drugs can aggravate the mental burden of patients and affect their prognosis [3]. At present, many psychotherapy techniques have been applied in the treatment of schizophrenia, which is of great significance for controlling symptoms, improving treatment compliance, and improving the social function of patients [4, 5]. However, existing psychotherapeutic techniques have a single intervention and lack holistic and comprehensive intervention methods [6]. Social cognitive interaction training (SCIT) is a therapy hypothesis developed by Roberts in 2007, which holds that the cognitive impairment caused by schizophrenia is separated into three parts: emotional perception, theory of mind, and attribution mode. As a result, the intervention for patients should provide holistic therapy from all three perspectives in order to significantly enhance patients' social cognitive performance [7]. At present, this treatment has been applied in a number of studies, but there are inconsistent reports on its therapeutic effect. The results of the study by Rocha et al. [8] showed that SCIT was effective in improving attribution bias and social function in patients. But another study by Dark et al. [9] showed that SCIT did not show any additional benefit in social cognition improvement compared with conventional treatment methods. In order to address the inconsistencies between different studies and to understand the important role of SCIT for the improvement of the prognosis of patients with schizophrenia, we performed this meta-analysis on the basis of the existing published literature.

The implementation of this quantitative meta-analysis is guided by the PRISMA recommended guidelines (the Preferred Reporting Items for Systematic Reviews and Meta-Analyses).

## 2. Method

### 2.1. Inclusion and Exclusion Criteria for Studies

The inclusion and exclusion criteria related to this meta-analysis were as follows: (i) subjects: all subjects were hospitalized patients with confirmed schizophrenia, without limiting that patients were in the first attack, relapse, and remission stages. To avoid heterogeneity, we excluded studies whose subjects were discharged patients in the rehabilitation stage. (ii) Grouping and control: all patients were divided into the intervention group and control group. Randomization sequence and allocation concealment study were preferred. Baseline data were compared between the two groups. (iii) The intervention group: on the basis of conventional drug therapy, social cognitive interaction training (SCIT) was given. (iv) Control group: routine medication and routine care were given, and studies with other specific methods, such as training in affect recognition (TAR) [10], were excluded from the control group. (v) Outcome indicators: PANSS score, negative symptom score, positive symptom score, and social function score after treatment were the main outcome indicators. (vi) Study type: included studies are quasirandomized controlled studies or cohort studies.

RETRACTED

### 2.2. Literature Search Strategy

We focused on the databases PubMed (https://pubmed.ncbi.nlm.nih.gov/), WOS (https://www.webofscience.com/), Scopus (https://www.scopus.com/), China National Knowledge Infrastructure (CNKI, https://www.cnki.net), and Weipu (https://www.cqvip.com/), a comprehensive and systematic search was performed, and all articles were published before April 2022. The search was performed by two researchers using a keyword free search mode with keywords including (“*social cognitive interaction training*” OR “*SCIT*” OR “*cognitive behavioral social skills training*” OR “*CBSST*”) AND (“*schizophrenia*”).

### 2.3. Selection of Literatures

Two researchers exported the retrieved articles from each database in a format that EndNote could identify, such as PubMed export suffix “*.Nbib*” and other databases' file storage with “.*ris*” suffix. All the retrieved literatures were imported into EndNote management, and the repeated literatures were removed by using the “repeated literature identification” function of the software. According to the established inclusion and exclusion criteria, two researchers read the title and abstract of the literature one by one to complete the screening of most of the articles. After screening the remaining articles on the Internet (or directly contacting the original author), receive the full text of the articles, read the full text of the articles, further screen, and obtain the final collection of included articles. If there was a disagreement regarding whether or not to include a particular piece, a third person was requested to make a decision.

RETRACTED

### 2.4. Data Extraction

The researchers obtained the data required for meta-analysis from the included literatures and recorded it in a tabular form. Data included gender ratio, mean age, initial PANSS score (mean ± variance), education level (%), residence, family psychiatric history, name of the published journal, first author, study region, study type, random sequence generation method, and outcome data of included patients. If the data of the study is not provided, it was marked as NR (not reported).

### 2.5. Literature Quality Assessment and Risk of Bias

Cochrane risk of bias 2.0 [11] was used to evaluate the risk of bias of the included studies, including 6 levels, and each level was given “low,” “some concern of risk,” and “high” for risk evaluation.

### 2.6. Statistical Methods

(i) Effect sizes: since different literatures may adopt different scales for the evaluation of the same indicator, we use standard mean difference (SMD) and 95% CI as effect size for the analysis of outcome indicators (except PANSS total score) and mean difference (MD) and 95% CI as effect size for PANSS total score. (ii) Heterogeneity test: for the heterogeneity of literatures displayed during analysis, we expressed it as tau^2^, and standard error (SE), *I*^2^, and *Q* tests were used for the test of heterogeneity; *I*^2^ > 50% or *P* < 0.1 indicated that the heterogeneity was not statistically significant, and there was heterogeneity between literatures. (iii) Effect model selection: random effects mode was used for analysis. (iv) Analytical tools: the analysis was completed using the R language toolkit metafor released by Cran-Project to present the analysis results in a forest plot. (v) Heterogeneity survey: metaregression analysis, the radial plot or Galbraith plot, and normal quantile-quantile (QQ) plot were used to analyze publication bias. (vi) Publication bias analysis: publication bias was analyzed by funnel plot and Egger's test, and Pr > |*z*| < 0.05 was considered statistically significant.

## 3. Results

### 3.1. Literature Screening Process and Results

The identification, screening, and inclusion process according to PRISMA regulations is shown in Figure 1. In this study, 692 literatures were initially searched, 266 were searched by PubMed, 136 were searched by WOS, 49 were searched by Scopus, 126 were searched by CNKI (Chinese), and 115 were searched by Weipu. After all literatures were imported into EndNote, a total of 98 repeated literatures were repeatedly judged. After removing the repeated literatures, the remaining 594 literatures were initially screened, non-RCT studies (176 literatures) and nonschizophrenia patients (25 literatures) were excluded. After inappropriate intervention methods (75 literatures), the remaining 318 literatures were included in the usability analysis; the full text could not be obtained in 76 literatures. The literatures without outcome indicators and with unusable data were further excluded. Finally, 14 literatures [8, 9, 12–23] were included.

RETRACTED

### 3.2. Basic Characteristics of Literatures

A total of 1167 patients with schizophrenia were included in this study, and all studies were RCT studies, including 590 patients treated with SCIT and 577 patients treated with TAU. There was 1 literature [12] on children (aged <18 years), and the remaining study subjects were all adult patients; the intervention duration ranged from 4 to 36 weeks, as shown in Table 1.

### 3.3. Quality Assessment of Literature

Figure 2 summarizes the details of methodological assessment of eligible studies assessed according to the Cochrane ROB 2.0. The overall quality of the 14 studies included in this study was good, with 0 articles (0.00%) for “high risk of bias,” 8 articles (57.14%) for “low risk of bias,” and 6 articles (42.86%) for “some concern of risk.” The results of the Cochrane ROB 2.0 confirmed that there was no significant bias in this meta-analysis.

### 3.4. Meta-Analysis Results

#### 3.4.1. Comparison of Negative Symptom Scores after Intervention

Among all 14 included studies, a total of 8 literatures [8, 12, 14, 15, 20–23] tried to compare SCIT with TSU for the comparison of negative symptom scores of patients with schizophrenia after treatment, the literatures [8, 14, 21, 22] were assessed by the SANS scale, and the literatures [12, 15, 20, 23] were assessed by the negative symptom subscale of PANSS scale. In the analysis, it was found that there was significant heterogeneity between the literatures (tau^2^ = 0.7979 (SE = 0.4864), *I*^2^ = 92.62%, Cochran *Q* test, *P* < 0.0001). The pooled ES obtained using the random effects model was SMD = −1.66 (95% CI (-2.32, -1.00), *P* < 0.0001), suggesting that patients had lower negative symptom scores after SCIT than after TSU treatment. A forest plot of pooled effects is shown in Figure 3.

#### 3.4.2. Positive Symptom Score after Intervention

Among all 14 included studies, a total of 4 literatures [8, 15, 20, 22] tried to compare the positive symptom scores of SCIT and TSU for patients with schizophrenia after treatment. All literatures were assessed by the positive symptom subscale of PANSS scale. The analysis found that there was significant heterogeneity between the literatures (tau^2^ = 12.878 (SE = 11.395), *I*^2^ = 96.91%, Cochran *Q* test, *P* < 0.0001). The pooled ES obtained using the random effects model was MD = −4.03 (95% CI (-7.69, -0.36), *P* = 0.03), suggesting that patients had lower positive symptom scores after SCIT than after TSU treatment. Forest plots of pooled effects are shown in Figure 4.

RETRACTED

#### 3.4.3. PANSS Total Score after Intervention

Among all 14 included studies, a total of 5 literatures [8, 12, 15, 20, 23] tried to compare SCIT with TSU for the PANSS total score after treatment in patients with schizophrenia, and significant heterogeneity was found between the literatures in the analysis (tau^2^ = 41.63 (SE = 34.21), *I*^2^ = 91.30%, Cochran *Q* test, *P* < 0.0001). The pooled ES obtained using the random effects model was MD = −6.33 (95% CI (-12.43, -0.23), *P* = 0.02), suggesting that the PANSS total score was lower in patients after SCIT than after TSU treatment. A forest plot of pooled effects is shown in Figure 5.

#### 3.4.4. Social Function after Intervention

Only 8 articles [8, 12, 15, 17, 18, 20, 23] attempted to compare the effects of SCIT with TSU on posttreatment social functioning in patients with schizophrenia, and significant heterogeneity was found between the articles in the analysis (tau^2^ = 0.257 (SE = 0.193), *I*^2^ = 82.15%, Cochran *Q* test, *P* < 0.0001). The pooled ES obtained using the random effects model was SMD = 0.77 (95% CI (0.34, 1.20), *P* < 0.001), suggesting that the social function of patients was improved after SCIT compared with TSU treatment. A forest plot of pooled effects is shown in Figure 6.

#### 3.4.5. Heterogeneity Survey

*(1) Regression Analysis*. This meta-analysis tried to find whether “age” was the result affecting the negative symptom score after treatment, and the results showed that *P* > |*t*| = 0.553; age was not the source of heterogeneity, as shown in Figure 7.

*(2) Radial Plot*. The comparison of negative symptom scores after treatment was shown by radial plot, and it can be seen from the presentation that all 8 articles were within the range without significant deviation, as shown in Figure 8.

*(3) Normal Quantile-Quantile (QQ) Plot*. The comparison of negative symptom scores after treatment was shown by the QQ plot, and it showed that 8 articles were within the range and without significant deviation, as shown in Figure 9.

#### 3.4.6. Analysis of Publication Bias

In the publication bias for the comparison of negative symptom scores after treatment, the funnel plot showed that the 8 literatures showed uneven distribution on both sides of the funnel, possibly with bias; however, in the quantitative analysis using Egger's test, *P* > |*t*| = 0.660, suggesting that there was no statistically significant publication bias, as shown in Figures 10 and 11.

RETRACTED

## 4. Discussion

SCIT is a comprehensive psychotherapeutic approach based on improving emotional perception, attribution style, and theory of mind ability in patients with schizophrenia [24]. Unlike existing cognitive theories, this approach focuses treatment on three categories of social cognition [25]. The results of existing clinical studies have shown that SCIT can significantly improve the emotional cognition, suggestion, and attribution methods of patients, thereby reducing the aggressive behavior of patients, improving the cognitive flexibility of patients, enhancing the needs of intimate relationships, and improving the social relationships of patients [26, 27]. In the study by Rocha et al. [8], SCIT improved these indicators compared with conventional treatment, as patients' cognitive bias, emotion recognition, theory of mind, and social perception were measured before and after treatment.

As the core symptom cluster of schizophrenia, negative symptoms are the main cause of protracted course and mental disability, and their occurrence is closely related to the abnormal cognitive pattern of patients to negative life events [28]. Patients generally tend to attribute multiple symptoms to the outside world, especially others in the outside world [29]. SCIT focuses on the correction of patient's unreasonable cognition, encourages patients to self-expose their emotions, ideas, and behaviors, guides patients to develop in an objective and correct direction when thinking about problems, improves patients' ability to solve realistic problems by changing patients' views and attitudes about people or things, and reduces patients' negative symptoms from the perspective of improving social cognition [30]. Although some studies [23] suggested that SCIT did not improve the negative symptoms of patients, the results of this pooled analysis showed that SCIT had a lower negative symptom score than TSU treatment (SMD = −1.66, 95% CI (-2.32, -1.00), *P* < 0.0001). The severity of negative symptoms is positively correlated with the degree of emotional cognitive deficits shown statically, and apathy, diminished volition, interest, or social impairment among negative symptoms may reduce the patient's theory of mind ability and make the patient's social experience accumulate less [31]. In SCIT training, patients are guided to share their own life examples, to bring patients to real social events, to continuously enrich their inner experience in sufficient discussion and practice role exchange, to cultivate the ability of patients to stand at each other's perspective in social communication to think about problems, to improve the patient's theory of mind level, to activate subjective initiative, and to continuously improve the patient's emotion [22].

RETRACTED

Furthermore, the combined findings of this research revealed that the positive symptom score and PANSS total score of patients after SCIT were lower than those following TSU therapy, indicating that SCIT treatment was helpful to the patient's illness recovery. Presumably, it is successful in alleviating positive symptoms in individuals with schizophrenia spectrum disorders, particularly delusions, by explaining what delusions are, describing the numerous possibilities of event occurrence, and differentiating facts from hypothesis through images and videos [14].

In the 8 literatures included in this study, we tried to compare the effect of SCIT and TSU on the social function of patients with schizophrenia after treatment. The pooled ES was SMD = 0.77 (95% CI (0.34, 1.20), *P* < 0.001), suggesting that the social function of patients after SCIT is improved compared with TSU. As a systematic social skills training, SCIT integrates behavioral therapy with behavior modification techniques, contains a large number of basic social skills such as eye contact, facial expression, sound size, and fluency of language, provides patients with sufficient practice opportunities, guides patients to adopt new social skills for emotional communication with others, reminds patients to make appropriate behaviors on different occasions to reduce frustration, and continuously obtains positive feedback from peers, which qualitatively corrects and improves patients' behaviors and improves patients' social skills [16]. SCIT's intervention process also employs the concept of team therapy, allowing patients to experience the strength of being accepted and supported, activating patients' ability to be interested in the surrounding things and thus reducing negative coping styles, improving patients' enthusiasm to participate in occupational therapy, and significantly improving patients' psychological and social functions [19]. The results of Hooker et al. [32] showed that the positive effect of SCIT on social cognitive skills may arise from its altered patient neural activity mechanisms.

The patients included in this study were all inpatients and did not include any community schizophrenic patients with stable disease. Roberts et al.'s study [33] attempted to apply this treatment to discharged patients and found that SCIT may be a promising intervention for community institutions that can serve psychiatric patients seeking to improve social functioning. In a Japanese study [34], it was shown that the application of SCIT in the community was feasible and tolerated by patients. Based on the improvement of social function in patients with mental illness, SCIT can be applied not only to patients with schizophrenia but also to patients with other mental illnesses such as autism and bipolar disorder [35, 36]. It has recently been shown that the human microbiome also has some influence on mood. Therefore, drugs capable of modulating the human microbiota, for example, amoxicillin [37] and ornidazole [38], also deserve attention.

RETRACTED

Although the general quality of the included literatures in this research was excellent, there was no substantial publication bias, and the radial plot and normal quantile-quantile plot indicated stable findings; it should be noted that this meta-analysis had limitations. For starters, there was clear variability among the literatures. We tried to explore the source of heterogeneity and found that the length of intervention did not affect the results. The heterogeneity of literatures may be related to that the patients included in different studies had different disease types and age levels and may also be related to different intervention methods implemented in each study (different therapeutic drugs, differences in the methods implemented by SCIT) or related to different scales used for outcome measurement. Because of numerous factors, we could not analyze them one by one. Second, there were too few included articles and only eight reports on negative symptom indicators, which may cause insufficient study data. Finally, we did not have group discussions on different countries and regions. Therefore, studies on this topic require more homogeneous, good-quality RCT literature to continue to be explored in depth.

Despite some limitations, the results of this meta-analysis support that SCIT helps to improve the relief of symptoms and the improvement of social function in patients with schizophrenia. However, more research is still needed to be deeply explored.

## Figures and Tables

**Figure 1:** The selection flow chart following PRISMA.

**Figure 2:** Summary plot of literature bias analysis.

**Figure 3:** Comparison of negative symptom scores after treatment between the two groups.

**Figure 4:** Comparison of PANSS positive symptom scores after treatment between the two groups.

**Figure 5:** Comparison of the PANSS total score after treatment between the two groups.

**Figure 6:** Comparison of social function scores after treatment between the two groups.

**Figure 7:** Regression analysis by age factor.

**Figure 8:** Radial plot.

**Figure 9:** Normal quantile-quantile (QQ) plot.

**Figure 10:** Publication bias: funnel plot.

**Figure 11:** Publication bias: Egger's quantification.

**Table 1:** Basic characteristics of the included studies.

First author, year	Observation group (SCIT)		Control group (TAU)		Population (O/C)	Duration of intervention	Outcome indicators
	M/F	Age	M/F	Age			
Rocha et al., 2021 [8]	5/1	29.5 ± 13.38	5/0	27 ± 6.12	6/5	20 weeks	(a)(b)(c)(d)
Dark et al., 2020 [9]	46/15	36.1 ± 10.7	40/19	37.5 ± 10.1	61/59	12 weeks	(d)(e)
Li et al., 2020 [12]	54/52	16.11 ± 1.44	55/47	16.13 ± 1.43	106/102	24 weeks	(a)(b)(c)(d)
Gordon et al., 2018 [13]	7/14	19-55	5/10	19-54	21/15	10 weeks	(e)(g)
Wang et al., 2019 [14]	20/10	26.4 ± 9.7	20/10	27.1 ± 8.5	30/30	4 weeks	(a)(f)
Zhang et al., 2019 [15]	32/26	42.5 ± 9.2	31/29	42.6 ± 8.1	58/60	9 weeks	(a)(b)(c)(d)
Tao et al., 2011 [16]	20/18	37.1 ± 11.5	18/20	39.0 ± 11.8	38/38	6 weeks	(d)(g)
Roberts et al., 2014 [17]	22/11	40.0 ± 12.2	22/11	39.4 ± 12.8	33/33	20 weeks	(d)(e)(g)
Wang et al., 2013 [18]	12/10	43.86 ± 11.65	8/9	40.88 ± 10.15	22/17	20 weeks	(d)
Lian et al., 2017 [19]	38/16	31.7 ± 8.2	36/15	33.0 ± 7.5	54/51	4 weeks	(g)
Shen et al., 2018 [20]	25/20	27.96 ± 7.66	21/24	31.06 ± 9.76	45/45	10 weeks	(a)(b)(c)(d)(g)
Mahmood et al., 2021 [21]	9/17	47.73 ± 11.36	50/50	53.24 ± 7.35	13/16	12.5 weeks	(a)(e)
Granholm et al., 2014 [22]	46/27	41.1 ± 10.4	53/23	41.6 ± 9.2	73/76	36 weeks	(a)(b)(e)
Xu et al., 2011 [23]	17/13	37.1 ± 14.9	17/13	35.6 ± 13.0	30/30	6 weeks	(a)(c)(d)

(a) Negative symptoms, (b) positive symptoms, (c) PANSS total score, (d) social function assessment, (e) social skills and performance, (f) rehabilitation efficacy, and (g) quality of life. M/F: male/female; O/C: observation/control; PANSS: positive and negative syndrome scale; TAU: treatment as usual.

RETRACTED

## Data Availability

The datasets used during the current study are available from the corresponding author on request.
